# High Glucose Activated Cardiac Fibroblasts by a Disruption of Mitochondria-Associated Membranes

**DOI:** 10.3389/fphys.2021.724470

**Published:** 2021-08-18

**Authors:** Ling-Yu Zhang, Rui-Ting Lin, Hao-Ran Chen, Yong-Cong Yang, Meng-Fei Lin, Lei-Gang Tian, Zhi-Qiong Pan, Lin Lin, Liang-Liang Zhu, Zhen-Jie Gu, Xue-Wen Chen, Yu-Jing Li, Shuai Chen, Shi-Yun Cai

**Affiliations:** Department of Cardiology, Maoming People’s Hospital, Maoming, China

**Keywords:** cell proliferation, glycolysis, mitochondria-associated membranes, signal transducer and activator of transcription 3, mitofusin-2

## Abstract

Cardiac fibrosis is evident even in the situation without a significant cardiomyocyte loss in diabetic cardiomyopathy and a high glucose (HG) level independently activates the cardiac fibroblasts (CFs) and promotes cell proliferation. Mitochondrial respiration and glycolysis, which are key for cell proliferation and the mitochondria-associated membranes (MAMs), are critically involved in this process. However, the roles and the underlying mechanism of MAMs in the proliferation of HG-induced CFs are largely unknown. The proliferation and apoptosis of CFs responding to HG treatment were evaluated. The MAMs were quantified, and the mitochondrial respiration and cellular glycolytic levels were determined using the Seahorse XF analyzer. The changes of signal transducer and activator of transcription 3 (STAT3) and mitofusin-2 (MFN2) in responding to HG were also determined, the effects of which on cell proliferation, MAMs, and mitochondrial respiration were assessed. The effects of STAT3 on MFN2 transcription was determined by the dual-luciferase reporter assay (DLRA) and chromatin immunoprecipitation (CHIP). HG-induced CFs proliferation increased the glycolytic levels and adenosine triphosphate (ATP) production, while mitochondrial respiration was inhibited. The MAMs and MFN2 expressions were significantly reduced on the HG treatment, and the restoration of MFN2 expression counteracted the effects of HG on cell proliferation, mitochondrial respiration of the MAMs, glycolytic levels, and ATP production. The mitochondrial STAT3 contents were not changed by HG, but the levels of phosphorylated STAT3 and nuclear STAT3 were increased. The inhibition of STAT3 reversed the reduction of MFN2 levels induced by HG. The DLRA and CHIP directly demonstrated the negative regulation of MFN2 by STAT3 at the transcription levels *via* interacting with the sequences in the MFN2 promoter region locating at about −400 bp counting from the start site of transcription. The present study demonstrated that the HG independently induced CFs proliferation *via* promoting STAT3 translocation to the nucleus, which switched the mitochondrial respiration to glycolysis to produce ATP by inhibiting MAMs in an MFN2-depression manner.

## Introduction

Diabetic cardiomyopathy extensively exists in patients with diabetes and poses a great health burden all around the world (Marfella et al., 2021). Cardiac fibrosis is the hallmark of diabetic cardiomyopathy (Bai et al., 2020; Peterson and Gropler, 2020). Moreover, unlike other primary diseases causing cardiac interstitial fibrosis, which are secondary to the primary cardiac insults, it has long been found that fibrosis in the ventricle could be evident in the situation without a documented cardiomyocyte damage during the development of diabetic cardiomyopathy (Regan et al., 1977). These indicated an “active” role of cardiac fibroblasts (CFs), which are the crucial effector cells in cardiac fibrosis, during the development of diabetic cardiomyopathy.

The CFs are capable of resisting apoptosis and preserve the potency to proliferate under unfavorable circumstances (Gottlieb, 2003; Mayorga et al., 2004). A wide range of mechanisms could be involved in this process, and mitochondria are believed to be the critical organelle in it (Bai et al., 2020). Mitochondria responds to various signals from the inner environment of the cells and regulates cell growth and death. Specifically, targeting the mitochondrial pathway-related apoptosis has been supposed to be effective in antifibrotic therapy (Kuehl and Lagares, 2018). Therefore, mitochondrial functions are of vital importance in cell proliferation, apoptosis, and fibrosis.

The regulation of mitochondrial function is complex, and several factors are involved. Among these factors, the mitochondria-associated membranes (MAMs), which refer to the sites of endoplasmic reticulum (ER)-mitochondria contacts, are critical. MAMs refers to a dynamic platform where ER tightly associates with mitochondria (Missiroli et al., 2018). MAMs are the pivotal structure for ER and mitochondrial cross talk, allowing the exchanges of intermediate metabolites and biological molecules to maintain cellular health and survival (Pinton, 2018). On the other hand, abnormal MAMs could cause cellular stress, dysfunction of calcium homeostasis, and inflammation that lead to cell death and disease development (Pinton, 2018).

Several critical molecules in maintaining MAMs have been identified, and mitofusin-2 (MFN2) is widely accepted as the important one (Hu et al., 2021). MFN2 is a mitochondrial protein that promotes mitochondrial fusion and maintains the mitochondrial-related network. MFN2 tethers ER and mitochondria and facilitates the establishment of MAMs (Annunziata et al., 2018). Under the diabetic condition, the expressions of MAMs and MFN2 are reduced in the heart, and this has been proposed as a therapeutic intervention for diabetic cardiomyopathy (Bach et al., 2005; Hu et al., 2019). Indeed, reinforcing MAMs *via* increasing the MFN2 expression has been proved to be a protective strategy for the damage of various organs caused by diabetes (Lopez-Crisosto et al., 2015).

However, the alterations of MAMs in CFs under diabetic conditions are rarely investigated. Given the importance of CFs in cardiac fibrosis triggered by diabetes, it is necessary to explore the detailed changes of MAMs in these effector cells. In the present study, we clarified the changes and underlying mechanisms of MAMs in CFs with the high-glucose treatment. Moreover, the expression of the critical molecule, MFN2, and the regulatory manner of its expressions, was also addressed.

## Materials and Methods

### Cell Cultures and Treatments

Human ventricular CFs were purchased from the ScienCell Research Laboratories (ScienCell, CA, United States) and maintained according to the instructions and previous reports of the manufacturer (Gao et al., 2020; Tao et al., 2021). Briefly, cells were cultured in the complete medium containing basic medium (fibroblast medium, FM-2; ScienCell) and supplements (10% fetal bovine serum, Gibco, CA, United States; fibroblast growth supplement-2, diluted to ×1 according to the instruction of the manufacturer, ScienCell; and 1% penicillin/streptomycin, Gibco) in the incubator at 37°C and 5% CO_2_. Cells were passaged when a confluence of 80% was reached, and cells in the passages of 6 and 7 were used for experiments in the current study.

For intervention, cells were treated with additional high glucose (HG) (50 mM, Sigma-Aldrich, MO, United States) or osmotic control (50 mM, mannitol, Sigma-Aldrich). To increase the MFN2 expression, the recombinant adenovirus carrying MFN2 coding sequences was used according to the previous report (Wang et al., 2021). Briefly, the shuttle plasmid, pDC315, was used to reconstruct the MFN2-expressing vector (pDC315-MFN2), and GFP was used as control. Ad-293 cells were co-transfected with the shuttle plasmids and adenovirus genomic plasmid pBHGlox^Δ^E13cre. Viruses were collected and amplified in 293A cells. Finally, cells were harvested and Adv were purified using the cesium chloride density gradient centrifugation approaches. For signal transducer and activator of transcription 3 (STAT3) inhibition, the small molecule compound specifically targeting STAT3 (Stattic, 10 μM; MCE, NJ, United States) was used.

### Assays of Cell Apoptosis and Proliferation

The apoptosis of CFs was assessed by using the flow cytometry method according to the previous report (Wu M. X. et al., 2021). Briefly, cells were collected and resuspended, which were subjected to staining with annexin V and propidium iodide using a commercially available kit according to the instruction of the manufacturer (Thermo Fisher Scientific, CA, United States). The fluorescence emission was detected using the fluorescein isothiocyanate and phycoerythrin channels. All the flow cytometry analyses were performed using the LSR Fortessa flow cytometer (Becton, Dickinson and Company, NJ, United States), and the data were analyzed by using the FlowJo software version 10 (Becton, Dickinson and Company, NJ, United States) according to previous report (Tao et al., 2021).

The cell proliferation was indicated by the Cell Counting Kit-8 (CCK-8) measurement according to the instruction of the manufacturer and previous report (Chen et al., 2020). Briefly, cells with different treatments were cultured in the medium with the CCK-8 reagent supplement. The absorbance of the supernatant was determined at 450 nm, and the data were recorded.

### MAMs Isolation

Mitochondria-associated membranes were isolated as described earlier (Tao et al., 2021). Briefly, CFs were ultrasonically fragmented, and cell debris were removed by low-speed centrifugation. Supernatants were collected and subjected to high-speed centrifugation, and pellets were obtained. The pellets were resuspended and subjected to ultrahigh-speed centrifugation, and the middle layers were carefully collected, which were subjected to another ultrahigh-speed centrifugation. The supernatants were removed, and the precipitants were used for protein quantification. The pure mitochondrial protein extracted using the commercially available kit (Thermo Fisher Scientific) was used as a control. The ratio of the protein contents (i.e., MAMs/mitochondria) represented the number of MAMs.

### Seahorse Assay and ATP Detection

The seahorse assays assessing the capacity of mitochondrial respiration indicated by the oxygen consumption rate (OCR) and assessing the glycolytic levels indicated by the extracellular acidification rate (ECAR) were performed according to previous report (Chen et al., 2020; Gao et al., 2020). The Seahorse XF Cell Mito Stress Test Kit (Agilent, DE, United States) was used to measure OCR, and the Seahorse XF glycolytic rate assay kit (Agilent) was used to determine ECAR. Briefly, cells were seeded in the Seahorse culture plate (Agilent) and the working medium (Agilent). Reagents were added, and OCR (or ECAR) was detected according to the instructions of the manufacturer.

The production of ATP was determined by using the commercially available kit according to the previous report (Wang et al., 2021). Briefly, cells were treated and supernatants were collected. Reagents were added according to the instructions of the manufacturer, and the absorbance was determined using a luminometer.

### Real-Time Quantitative Reverse Transcription Polymerase Chain Reaction and Western Blot

The real-time quantitative reverse transcription PCR (RT-qPCR) and Western blot were performed according to previous reports (Zhang et al., 2017; Guan et al., 2021). In brief, for RT-qPCR, cells were collected after removing the medium. The total RNAs were extracted by using the TRIzol methods, which were then subjected to reverse transcription using the commercially available kit. Finally, the PCRs were performed using the SYBR method in the LightCycler^®^ 480 (Roche, Basel, Switzerland). The data were analyzed using the 2^–ΔΔCT^ method, and the expressions of target genes were normalized to those of tubulin.

For Western blot, cells were collected, and total proteins were extracted. The sodium dodecyl sulfate-polyacrylamide gel electrophoresis was performed, followed by transfer to polyvinylidene difluoride (PVDF) membranes. Target PVDF membranes were collected and incubated with antibodies (MFN2, Abcam, Cambridge, United Kingdom) after blocking, which were then subjected to incubation with the enhanced electrochemiluminescence (Millipore, MA, United States) and visualized; the bands were observed and captured by using an imaging system (Bio-Rad, CA, United States). The optical density was analyzed using the Image J software (National Institutes of Health, MD, United States), and α-tubulin was used as the loading control.

To determine the intracellular distribution of STAT3, cytoplasmic, and nuclear proteins were isolated separately using the commercially available kit (NE-PER^TM^ Nuclear and Cytoplasmic Extraction Reagents, Thermo Fisher Scientific) according to the instruction of the manufacturer. The proteins were then subjected to Western blot for detecting the contents of STAT3.

### Analysis of MFN2 Gene Promoter, a Dual-Luciferase Reporter Assay (DLRA), and Chromatin Immunoprecipitation (CHIP)

To identify the potential sequences targeted by STAT3, the MFN2 gene promoter sequences reported by the previous study (Sorianello et al., 2012) were analyzed by using the JASPER formula (Fornes et al., 2020). The DLRA and CHIP were performed according to the previous report (Zhang et al., 2017). For DLRA, the reconstructed pGL4.23 enhancer (Promega, WI, United States) containing the −1,982 bp and +45 bp counting from the transcription start site of MFN2 according to the previous report (Sorianello et al., 2012) and the thymidine kinase promoter-Renilla luciferase reporter plasmid were co-transfected into the CFs. Later, cells were collected, and the luciferase activity was determined using the fluorescence spectrophotometer according to the instruction of the manufacturer (Promega). To identify the core sequence within the abovementioned −2,027 bp in the regulation of MFN2 transcription, different segments of MFN2 promoter sequences were constructed. The pGL4.23-enhancer vector without carrying any MFN2 sequence was used as the mock control.

The CHIP with the STAT3 antibody was performed using the Pierce Agarose ChIP Kit (Thermo Fisher Scientific) according to the previous report (Zhang et al., 2017). Briefly, supernatants were removed, and cells were cross-linked by using formaldehyde. Then, cells were lysed and sonicated to generate DNA fragments. Supernatants were collected and subjected to immunoprecipitation using the STAT3 antibody (Abcam) to obtain the DNA-protein complex. DNAs in the precipitated complex were recovered and extracted for the qPCR detection. The sonicated lysates before immunoprecipitation were used as the input control. Primers used for DLRA and CHIP were provided in Supplementary Table 1.

### Statistical Analysis

The data were expressed as mean ± SEM. The *t*-test was used to compare the mean difference between the group and the one-way ANOVA followed by which the Student–Newman–Keuls *post hoc* test was used if three groups were involved. All the statistical analyses were performed by using the OriginPro 2018 software program (OriginLab, MA, United States), and a *p*-value < 0.05 was considered statistically significant.

## Results

### HG Leads to Decreased Mitochondrial Oxidation but Increased Glycolysis, ATP Production, and Proliferative Ability

We first investigated the effects of HG on cell apoptosis and variability. According to the results from flow cytometry, HG did not affect apoptosis in the static situation (Figure 1A). Moreover, HG reduced the apoptosis of CFs when cultured in the serum-deprived medium (Figure 1B). Similarly, HG increased the cell variability as manifested in the results from the CCK-8 measurements (Figure 1C).

**FIGURE 1:** Effects of high glucose on cardiac fibroblasts apoptosis in static **(A)** or serum-deprived condition **(B)**, proliferation **(C)**, ATP production **(D)**, mitochondrial respiration **(E)**, glycolysis **(F)**, and mitochondrial potential **(G)**. *, compared with the control, *P* < 0.05; **, compared with the control, *P* < 0.01. Con, control; HG, high glucose; OD, optical density; ATP, adenosine triphosphate; OCR, oxygen consumption rate; ECAR, extracellular acidification rate; FCCP, trifluoromethoxy carbonylcyanide phenylhydrazone; Rot/AA, rotenone/antimycin A; 2-DG, deoxy-D-glucose.

Adenosine triphosphate production is one of the key factors supporting cell proliferation, and we next examined the changes of ATP produced by CFs cultured in HG. As shown in Figure 1D, HG increased the total ATP production. However, mitochondrial respiration, as assessed by the Seahorse XF analysis and indicated by the peak oxygen consumption, was moderately but significantly reduced on the HG treatment (Figure 1E). In contrast, cellular glycolytic levels, as indicated by ECAR, were dramatically increased in HG-treated cells (Figure 1F). Mitochondrial health is vital for maintaining its respiratory function, and mitochondrial membrane potential is reliable in assessing mitochondrial damage. We, therefore, continued to explore the changes in mitochondrial membrane potential. As shown in Figure 1G, CFs cultured in the HG medium displayed a slightly but statistically significant reduced mitochondrial membrane potential. All these results showed that HG facilitated energy production toward glucose metabolism, which mainly relied on glycolysis.

### HG-Induced Cell Proliferation and Glycolysis *via* the Reduction of MAMs in an MFN2-Dependent Manner

As MAMs are critically involved in hyperglycemia-induced pathological conditions, we continued to explore the alterations of MAMs in CFs under the HG treatment. As expected, HG resulted in reduced MAMs (Figure 2A). In accordance with this, MFN2 expression, either at the protein (Figures 2B,C) or mRNA level (Figure 2D), was significantly decreased in cells treated by HG.

**FIGURE 2:** Effects of high glucose on MAMs **(A)** and expression of MFN2 **(B–D)**. Effects of forced MFN2 expression on MAMs **(E)**, cell proliferation **(F)**, ATP production **(G)**, glycolysis **(H)**, and mitochondrial respiration **(I)**. ^#^, compared the HG + GFP, *P* < 0.05; ^##^, compared with the HG + GFP, *P* < 0.01. MAMs, mitochondria-associated membranes; MFN2, mitofusin-2. Other abbreviations are the same as Figure 1.

Despite that the reduction of MAMs and MFN2 levels were confirmed, the causality between these reductions and changes in cell proliferation, ATP productions, and mitochondrial respiration is still unknown. Therefore, we continued to clarify these relationships. The forced MFN2 expressions were performed to reconstruct MAMs in HG-treated CFs (Figure 2E). Results for the proliferation of MFN2-expressing CFs are shown in Figure 2F. As described earlier, MFN2 expression suppressed the CCK-8 contents, indicating an inhibitory effect on cell proliferation. In accordance with this, ATP productions were also decreased in MFN2-expressing cells (Figure 2G). Similarly, the glycolytic levels were decreased (Figure 2H), while mitochondrial respiration was increased in MFN2-expressing cells (Figure 2I). All these results showed that MFN2 downregulation and MAMs reduction play a key role in HG-induced cardiac proliferation.

### Nuclear STAT3, but Not Mitochondrial STAT3, Is Responsible for HG-Induced MFN2 Suppression

Although the mechanism of HG downregulating MFN2 is unknown, we continued to explore it. Since STAT3 is critically involved in HG-induced pathological conditions, we examined the alterations of STAT3. STAT3 is a dual-action factor, which could act as a transcription factor or a mitochondrial chaperone depending on the intracellular location. Unexpectedly, the mitochondrial STAT3 contents were not significantly different in cells treated with HG or control (Figures 3A,B). In contrast, the p-STAT3 levels were increased in HG-treated cells (Figures 3A,C). In accordance with this, STAT3 contents in the nucleus were also moderately increased (Figures 3A,D).

**FIGURE 3:** Effects of high glucose on subcellular STAT3 contents **(A–D)**. Effects of STAT3 inhibitor on MFN2 expression **(E–G)**. mt-STAT3, mitochondrial STAT3; VDAC1, voltage-dependent anion channel 1; p-STAT3, phosphorylated STAT3; t-STAT3, total STAT3; n-STAT3, nuclear STAT3; His-H, histone H. ^#^, compared with HG, *P* < 0.05; ^##^, compared with HG, *P* < 0.01. Other abbreviations are the same as Figure 1.

Signal transducer and activator of transcription 3 has been reported to negatively regulate MFN2 expression, and we continued to explore the role of STAT3 alteration in the regulation of MFN2 expression. STAT3 inhibitor, stattic, was used to inhibit the nuclear translocation, and the MFN2 expression was reassessed. As shown in Figures 3E–G, stattic significantly upregulated the MFN2 expression in either the protein (Figures 3E,F) or the mRNA (Figure 3G) level.

All these results consistently indicated that HG-induced MFN2 inhibition *via* the activation of STAT3.

### STAT3 Directly Suppressed MFN2 Transcription in the Presence of HG

The above results indicated that STAT3 may regulate MFN2 expression by the inhibition of its transcription, and we continued to confirm this hypothesis. First, the transcriptional inhibitor, actinomycin D (ActD), was used to observe the role of transcriptional mechanisms on HG-induced MFN2 suppression. As expected, ActD completely abolished the downregulated effects of HG on MFN2 expression (Figure 4A).

**FIGURE 4:** High glucose-induced STAT3 interacting with the MFN2 promoter and depressed its transcription. **(A)** Effects of transcription inhibitor, ActD, on MFN2 expression in the presence of high glucose. **(B)** Graphically illustrating potential STAT3-binding sites in MFN2 promoter predicted by using the JASPER formula. The darkness of color refers to the predicted score. Darker color indicates a high score. **(C)** Effects of high glucose and STAT3 inhibitor, stattic, on MFN2 promoter transcriptional activity. **(D)** Effects of MFN2 promoter segments on MFN2 promoter transcriptional activity in the presence of high glucose and STAT3 inhibitor. **(E)** Results of CHIP. ActD, actinomycin D; CHIP, chromatin immunoprecipitation; P2027, pGL4.23-(-2027); P425, pGL4.23-(-425); Ab, STAT3 antibody. Other abbreviations are the same as Figures 1, 3.

Then, the acknowledged MFN2 promoter sequences were analyzed, and the roles of potential STAT3-binding segments under HG conditions on MFN2 promoter transcriptional activity were directly analyzed using the DLRA. According to the results predicted from the JASPAR formula, a total of 14 putative STAT3-binding sites were identified, and sequences locating around the −400 bp (−394 to −404, 5′-CTACTAGAAAA-3′, and −410 to −420, 5′-CTTTTTAAAAA-3′, counting from the transcription start site of the reverse chain; Figure 4B) in the reverse chain were predicted to be the highest possibility in regulating the MFN2 transcription. As shown in Figure 4C, HG suppressed the MFN2 promoter activity, which could be counteracted by co-treatment with stattic. Moreover, segments around the abovementioned −400 bp showed a much more pronounced decreased luciferase activity upon HG treatment (Figure 4D). The CHIP using STAT3 antibody confirmed the binding of STAT3 and the core sequences (around −400 bp within the reverse chain) in the MFN2 promoter region in the HG treatment (Figure 4E).

All these results demonstrated that HG suppressed the MFN2 promoter activity in a STAT3-dependent manner, and the potential core sequences involved were located near the start site of transcription.

## Discussion

Cardiac fibrosis is the hallmark of diabetic cardiomyopathy, which could be evident without even in the situation that no obvious cardiomyocyte damage could be found. This indicated an “active” activation of cardiac fibroblast during this process. However, the mechanisms underlying are unknown. In the present study, we addressed the alterations of MAMs in cardiac fibroblast in HG condition and documented that the changes of MAMs, which are mediated by the STAT3/MFN2 mechanism, are the critical reason for the enhanced cardiac fibroblast proliferation in this situation.

Mitochondria-associated membranes refer to the contact sites of ER and mitochondria. It is a crucial subcellular structure for the communication of ER and mitochondria, which are important for cell growth and apoptosis, calcium homeostasis, substrates exchanges, autophagy, and lipid metabolism (Danese et al., 2017). It is well accepted that MAMs could be regulated by hyperglycemic/HG. A study in the diet-induced diabetic mice found that more MAMs but reduced calcium exchanges due to the increased MAMs thickness were observed in diseased mice (Dia et al., 2020). Moreover, reestablishing MAMs counteracted the damage of cardiomyocytes (Dia et al., 2020). In contrast, other studies reported significantly reduced MAMs under the diabetes condition (Yang et al., 2021). Recently, it is reported that diabetes and HG resulted in the decrease of MAMs in regulatory T cells, which affect cytokines production and indirectly affect cardiac fibroblast proliferation (Tao et al., 2021). According to the knowledge, less evidence could be available regarding cardiac fibroblast itself under HG condition. However, based on the conclusions from previous studies, it could be plausible to infer that different cell types may respond differently to HG treatment, and more studies are needed to explore details.

Mitochondria-associated membranes are dynamically and tightly regulated, and many molecules were involved in them (Townsend et al., 2020). Among these genes, many were also involved in the regulation of mitochondria. MFN2 is a gene facilitating mitochondrial fusion (Han et al., 2021). It inhibits mitochondrial fission and is being a target protein for mitophagy (Mengus et al., 2021). Despite no evidence reporting the association between diabetes and MFN2 in the cardiac fibroblast, it has been reported that MFN2 was reduced in diabetes condition in various cell types (Bach et al., 2005; Sebastian et al., 2012). In the present study, we showed that the re-expression of MFN2 reconstructed MAMs and facilitated mitochondrial respiration, making the cells produce ATP from oxidative phosphorylation instead of glycolysis. This restricts the rapid production of ATP and may, thus, slow down cell proliferation. The effects of MFN2 and the alterations of MAMs in this process are certainly notwithstanding; the precise role of MAMs should be interpreted in caution, which could be confounded by mitochondrial dynamics. The enhanced MFN2 expression increased the mitochondrial fusion while reducing fission, and this has been reported to decrease glycolysis during the cardiac fibroblast activation (Gao et al., 2020). Previous studies found that HG-induced mitochondrial fission in various cell types, (Kobayashi et al., 2020; Wu Q. R. et al., 2021) and these may further support the MAM-independent effects in the study. Therefore, it should be noted that the alterations of mitochondrial fusion and fission may independently induce mitochondrial respiration and inhibit glycolysis. Therefore, the increased mitochondrial respiration induced by MFN2 overexpression may be the result of the restoration of respiratory function, which may be MAM-dependent and -independent.

Some limitations of the current study should be acknowledged. First, the effects of HG on CFs were not verified *in vivo*, resulting in that no *in vivo* data could be available in illustrating this issue. Second, we did not investigate other molecules involved in the regulation of MAMs. As mentioned above, MFN2 could independently promote mitochondrial fusion. This makes it difficult to clarify the precise role of MAMs in the alterations of respiratory function, glycolysis is actually caused by MFN2 overexpression, and the potential role of mitochondrial fusion itself could not be ruled. Finally, the current study focuses on MAMs in HG-induced cardiac fibroblast proliferation, and other mechanisms [e.g., mitochondrial biogenesis also has been reported to be induced by HG in other cell types (Yan et al., 2018)] are not involved.

Despite the limitations, the current study demonstrated that HG independently and directly caused cardiac proliferation. Detailed mechanisms involved in STAT3- and MFN2-induced MAMs regulation were addressed. There is a need to carry out *in vivo* study to give more robust evidence showing the effects of diabetes on cardiac fibroblast. Moreover, there is a greater need for studies on mechanisms involving more critical molecules than is now customary to provide more details revealing the development of cardiac fibrosis in diabetic cardiomyopathy.

## Data Availability Statement

The original contributions presented in the study are included in the article/Supplementary Material, further inquiries can be directed to the corresponding author.

## Author Contributions

L-YZ, R-TL, H-RC, Y-CY, and M-FL designed and performed the experiments, and collected and analyzed the data. L-GT, Z-QP, LL, L-LZ, Z-JG, and X-WC helped to performed the experiments and collected the data. L-YZ, R-TL, and H-RC completed the manuscript. L-YZ, X-WC, Y-JL, SC, and S-YC analyzed the data and illustrated the figures. All authors contributed to the article and approved the submitted version.

## Conflict of Interest

The authors declare that the research was conducted in the absence of any commercial or financial relationships that could be construed as a potential conflict of interest.

## Publisher’s Note

All claims expressed in this article are solely those of the authors and do not necessarily represent those of their affiliated organizations, or those of the publisher, the editors and the reviewers. Any product that may be evaluated in this article, or claim that may be made by its manufacturer, is not guaranteed or endorsed by the publisher.
